# Signal-to-Noise Ratio Comparison of Several Filters against Phantom Image

This article has been retracted.

**DOI:** 10.1155/2022/4724342

**Published:** 2022-03-26

**Authors:** Muhammad Hameed Siddiqi, Yousef Alhwaiti

**Affiliations:** College of Computer and Information Sciences, Jouf University, Sakaka, Aljouf 2014, Saudi Arabia

## Abstract

Image denoising methods are important in order to diminish various kinds of noises, which are presented either capturing the image or distorted during image transmission. Signal-to-noise ratio (SNR) is one of the main barriers which avoids the theoretical observations to be accomplished in practice. In this study, we have utilized various kinds of filtering operators against three various noises, which are the signal-to-noise ratio comparison against the phantom image in spatial and frequency domain. In frequency domain, the average filter is used to smooth the image and frequency domain, and Gaussian low-pass filter is applied with empirically determined cutoff frequency. This work has six major parts such as applying average filter, determining the SNR of region of interest, transforming the image in frequency domain by discrete Fourier transform, obtaining the rectangular Gaussian low-pass filter along with a cutoff frequency, multiplying them, and carrying out the inverse Fourier transform. These steps are repeated accordingly until the resulting image SNR is equal to or greater than the spatial domain SNR. In order to achieve the goal of this study, we have analyzed the proposed approach against some of complex phantom images. The performances of these filters are compared against signal-to-noise ratio.

## 1. Introduction

Signal-to-noise ratio (SNR) has a significant role in many research fields such as signal and image processing, computer vision, artificial intelligence, and machine learning. Occasionally, SNR might be the main barrier which avoids theoretical observations to be accomplished in practice. Conservative filtering and optimization methods [1] are the general techniques for SNR enhancement. Commonly, the Gaussian filtering technique is more effective but less efficient, and the regularization technique is more efficient but less effective. Moreover, SNR is utilized to illustrate the quality of image. Basically, the sensitivity of the imaging approach is explained in the terms of the signal level that yields a threshold level of SNR. In imaging approaches, the image quality enhancement and noise reduction are the major steps. Image denoising efficiently conserves the edges of the image to a higher range in the smooth areas [2].

Image denoising is a significant process for reinstating the noise-free pictures from the noisy annotations which aid in conserving the texture and edges located in the corresponding pictures [3, 4]. Image denoising is measured as an important stage in color examination, segmentation, and feature extraction and selection [5]. There are lots of denoising approaches presented for diminishing noise from the various images.

A state-of-the-art approach was proposed by [6] for denoising which increases the image resolution through a model network assessed on identical data. First, this approach extracted the frames from video clips and then screened them using a trigonometric-Gaussian operator to reduce noise from the image. After this, the adaptive histogram equalization was employed in order to revise the contrast of the image that finally improved the resolution of the image [6]. However, the major limitation of adaptive histogram equalization is the propensity to over-intensify noise in comparatively homogeneous image areas [7]. Similarly, an adaptive and efficient method was proposed by [8] for image denoising, where they utilized the updated version of cuckoo search approach. In this method, two-sided filtering noisy image is enhanced through unsharp window and then utilized as the supervision image for the developed optimum supervised filtering method. However, the cuckoo searching method has the clear phenomenon of the early conjunction issue that is simply stuck into local optimum [9].

Therefore, the contribution of this study is described as

(i) This study compares the signal-to-noise ratio of a phantom image in spatial and frequency domain.
(ii) In frequency domain, average filter is utilized to smooth the picture and frequency domain, and Gaussian low-pass filter is applied with empirically determined cutoff frequency.
(iii) This work has five major parts:
  1. Apply average filter
  2. Determine the SNR of region of interest
  3. Transform the image in frequency domain by discrete Fourier transform
  4. Obtain the rectangular Gaussian low-pass filter along with a cutoff frequency
  5. Multiply them and do the inverse Fourier transform.
(iv) These steps are repeated accordingly until the resulting image SNR is equal to or greater than the spatial domain SNR.
(v) (v)In order to achieve the goal of this study, we have analyzed the proposed approach against some of complex phantom images.

The remaining article is arranged as follows.  Section 2 prescribes a comprehensive literature review against the proposed approach.  Section 3 explains the details of the proposed methodology.  Section 4 presents the performance evaluation of the developed approach against phantom images. Finally, the study is concluded with some forthcoming directions in Section 5.

## 2. Literature Review

Image denoising is a significant process for reinstating the noise-free pictures from the noisy annotations which aid in conserving the texture and edges located in the corresponding pictures. The authors of [10] developed an integrated method for image denoising. In this system, they combined two-dimensional disparity decomposition and nonlocal reprojection methods, in which the corresponding image is decomposed into a series of variational mode functions to make the denoising step easier. However, this approach considered synthetic images for validation that cannot be employed in real domains. Likewise, in [11], the authors introduced a new framework for image denoising. This framework has the ability to separate the signals from noise through a learning set of renovation in the feature space. After the separation, the denoising might be attained by choosing the conforming base of the signal subspace and projecting the input into such space. However, they lost much information during the separation process that make the denoising process a challenging task. Furthermore, the authors of [12] performed a correlative examination of various noise removal techniques against different operators in spectral images. These images are presented with various kinds of noise and further operators are employed to denoise the corresponding image. They utilized different group of filters such as Gaussian filter, Prewitt filter, Wiener filter, and Sobel filter for denoising. However, Prewitt and Sobel filters are sensitive to noise in edge detection and orientation, which means that if we increase noise of the image, then the accuracy will be decreased [13].

On the other side, different denoising methods such as nonlocal mean operator, wavelet transform, and median operator were proposed by [14, 15]. In their experiments, they added various types of noises such as Gaussian, salt and pepper, and speckle noise on X-ray and MRI images. However, these filters not only smooth the data to diminish noise but also blur the corresponding edges of the image as well [16]. A multilayered wavelet transform-based methodology was investigated by [17] for denoising under the presence of crop images. In their wavelet-based algorithm, they ignored low-frequency coefficients, while expanded high-frequency coefficients on, respectively, horizontal, vertical, and diagonal directions. However, wavelet transform has one of the common disadvantages such as poor directionality and shift invariance [18]. Similarly, in [19], the authors proposed a new deep generative network coupled with several target images and adaptive termination situation. They generated two clear target images by using a normal denoising technique that enabled best guidance during conjunction step and improved its speed. However, this approach suffered from overfitting problem.

An integrated method in [20] was based on the combination of bilateral operator and anisotropic diffusion method. This method performed the smoothing of the homogeneous areas without disturbing the edges of the corresponding image. However, the bilateral filter does not provide good results at higher noise levels. Also, one of the general limitations of the anisotropic diffusion method does not have the ability to preserve the shrill edges and details of the denoised image [21]. Similarly, the authors of [22] proposed a data augmentation technique in order to resolve the problem of overfitting that was due to the absence of the truth image. However, this approach is not applicable in real-world domains because of low processing speed. A multilevel wavelet transform was proposed by [23] for the image denoising that was distorted by selecting the horizontal coefficients for processing, which was based on tri-state median and switching median operators, respectively. Different types of rules were employed for each operator against various levels of salt-and-pepper noise. However, wavelet transform has one of the common disadvantages such as poor directionality and shift invariance [18].

A recent work has been presented by [24], which exposed a missing edge in order to integrate various approaches. The main advantage of this approach is to process the image without preprocessing step to find the mode of the following distribution. However, this approach works only in controlled environment. Likewise, a new integrated denoising system was proposed in [25], where they utilized various kinds of evaluation metrics such as structural similarity index measure, mean square error, contrast to noise, signal-to-noise ratio, and cross correlation. However, the image structure data might not properly be preserved by these noising methods [26]. Similarly, a latest denoising method was proposed [27] that relied on immoral images alone for approach training. It is an unsupervised technique which employed a design of blind-spot network. It needs only a single noisy image as its input and, hence, is well-matched for medical settings. However, this approach needs the accessibility of pairs of noisy images, and the gaining of these pairs along with some constants is only possible for static domains [28]. A robust method was designed by [29] for CT image denoising, which was the combination of various filters such as Gaussian and median filters. The effect of the shadow from CT images was removed by employing the Sobel method that detected the pixels of the edges and then assigned them to grain stages based on threshold. However, this approach does not efficiently work when the noise of spatial density is high [30].

An edge aware denoising method was recommended by [31] in order to get the goal of conserving the material of the original picture when utilizing the features of the noisy picture. However, this approach has a generalized issue such as weak antinoise capacity and false edge [32]. Another denoising scheme was developed in [33] that was based on different wavelet transforms against the threshold value. They selected the threshold value and wavelet structure with the help of spatial adaptivity and hybrid techniques, respectively. However, the wavelet transform has one of the common disadvantages such as poor directionality and shift invariance [18]. Moreover, this scheme is heuristic because of the manual selection of threshold. On the contrary, a deep neural network-based model was proposed in [34, 35] in order to observe the quality of the image from the denoising of a complete viewpoint of the CT image. In their respective work, first, they generated a library having innovative denoising styles of deep neural network. This library was included of denoising styles that was demonstrated and trained one by one to predict the best performance. However, this method showed some concerns such as complex optimization and computational expenses during denoising [36]. Similarly, a Haar wavelet transform-based method was developed in [37] for image denoising. First, analyze the memory necessities of the algorithm and computational complexity. To improve the significance, an integration of the convolution and recursion methods are utilized in order to understand the Haar filter bank, and gradient ancestry technique is employed to determine the reduction factors. However, the main limitation of the Haar wavelet transform is the features' disjointedness which leads to problems for simulating continuous signals [38]. Likewise, the authors of [39, 40] employed statistical features in order to diminish the noise from the image; however, their performances degrade against naturalistic domains.

## 3. Proposed and Ensembled Denoising Approach

In the proposed approach, we utilized various kinds of operators for denoising. The overall flow diagram is presented in Figure 1.

### 3.1. Averaging Filter

Averaging filter is diminishing the total intensity differences among the pixels. Generally, the averaging filter is used to substitute the value of every pixel within an image based on the average value of its surroundings, which has the effect of removing the value of the pixels that are misleading of their neighbors. For this filter, the template functions are the union such that 1/9 to confirm that the output of averaging nine white pixels is white but not in excess of white. It depends on the window that presents the size and shape of the region for the expected sample during the mean estimation. In this filter, 3 × 3 square mask is utilized as described in Figure 2.

For a common execution, we explained the size of the filter as “*W*_*S*_ is the size of window” and the size of template is *W*_*S*_ × *W*_*S*_. Then, we create the average of the entire pixels inside the region enclosed through the template, which is divided by the amount of points in the mask of the template. This is a straight execution of a common averaging filter instead of utilizing the convolution of the template filter as

(1) $$\begin{array}{c} A\left(I,W_{s}\right)≔\left|\begin{array}{c} \text{New}\leftarrow \text{zero}\left(I\right),\\ \text{Partial}\leftarrow \text{floor}\left(\frac{W_{s}}{2}\right),\\ \text{for }i\in \text{ Partial}..\text{Col}\left(I\right)-\text{Partial}-1,\\ \text{for }j\in \text{ Partial}..\text{Row}\left(I\right)-\text{Partial}-1,\\ {\text{New}}_{j,i}\leftarrow \text{floor}\left[\frac{\sum_{x=0}^{W_{s}}\sum_{y=0}^{W_{s}}I_{j+x-\text{Partial},i+y-\text{Partial}}}{W_{s}\times W_{s}}\right], \end{array}\right. \end{array}$$

where *I* is the corresponding image, *W*_*s*_ is the size of the window, and Col represents the number of the columns, respectively.

We need to design a template to execute the averaging filter by utilizing the convolution of the template filter, although the ease of the direct averaging filter typically prevents such types of executions. This diminishes the noise that is one the advantage of the averaging filter. However, the averaging filter may cause blurring that diminishes the features of the image. Therefore, we utilized Fourier transform to permit the components of the low frequencies and stop the components of the high frequencies.

### 3.2. Fourier Transform

The Fourier transform contains a set of *K* points *p*_*i*_ (tested through a frequency that is equal to the rate of testing) in the tested frequencies *F*_*pv*_ and is given as

(2) $$\begin{array}{c} Fp_{v}=\frac{1}{\sqrt{K}}\sum_{i=0}^{K-1}p_{i}e^{-j\left(2\pi /K\right)iv}. \end{array}$$

This explains the discrete correspondent Fourier transform that is substituted through a group of samples, the consecutive frequencies of the samples, and the summation of the frequencies. If the Fourier transform is applied to the pulse samples in a mask having range 0∼*K*/2–1, when the pulsation finishes, then equation (1) becomes as follows:

(3) $$\begin{array}{c} Fp_{v}=\frac{1}{\sqrt{K}}\sum_{i=0}^{k/2-1}Se^{-j\left(2\pi /K\right)iv}. \end{array}$$

The summation of the geometric evolution might be assessed as

(4) $$\begin{array}{c} \sum_{k=0}^{K}s_{0}r^{k}=\frac{s_{0}\left(1-r^{k+1}\right)}{1-r}. \end{array}$$

The sampled pulsation of the Fourier transform is given below:

(5) $$\begin{array}{c} Fp_{v}=\frac{S}{\sqrt{K}}\left(\frac{1-e^{-j^{\left(2\pi /K\right)\left(K/2\right)v}}}{1-e^{-j^{\left(2\pi /K\right)v}}}\right). \end{array}$$

Through reordering, we can obtain

(6) $$\begin{array}{c} Fp_{v}=\frac{S}{\sqrt{K}}e^{-j^{\left(\pi v/K\right)\left(1-2/K\right)}}\frac{\sin\left(\pi v/2\right)}{\sin\left(\pi v/K\right)}. \end{array}$$

Hence,

(7) $$\begin{array}{c} \left|Fp_{v}\right|=\frac{S}{\sqrt{K}}\left|\frac{\sin\left(\pi v/2\right)}{\sin\left(\pi v/K\right)}\right|, \end{array}$$

as the scale of the exponential is 1.

The spatial frequency is represented by the ratio of the pixels' intensity variations.  Figure 3 indicates various frequencies of an image, where the higher frequencies are focused throughout the axis distributing the image in quad. Higher frequencies are described by the attentions of high amplitude waves in small checker board outline; while, the bends have lesser frequencies that are described by large regions of closer constant points.

When we employed the digital images, the continuous function has never been utilized; however, we just considered a limited number of samples that are made by the number of pixels. In order to analyze an image, we need Fourier transform that is inherited from continuous FT and is represented by

(8) $$\begin{array}{c} H\left(u,v\right)=\frac{1}{MN}\sum_{x=0}^{M-1}\sum_{y=0}^{N-1}h\left(x,y\right)e^{-j2\pi \left(ux/M+vy/N\right)}. \end{array}$$

Equation (8) is converted to spatial domain and is represented by

(9) $$\begin{array}{c} h\left(u,v\right)=\sum_{x=0}^{M-1}\sum_{y=0}^{N-1}H\left(u,v\right)e^{j2\pi \left(ux/M+vy/N\right)}. \end{array}$$

It is obvious that both the processes of discrete Fourier transforms and inverse Fourier transforms are equivalent. Actually, the code which performs these processes might be the similar considering the route of the transform and accordingly sets up the symbol of the exponential.  Figure 4 shows an example of the Fourier transformed image.

### 3.3. Gaussian Low-Pass Filter

This filter describes the region from which we can collect spectral components, and the size of the region presents the range of the retained frequencies. If we collect the points from the center of the circular area and inverse Fourier transform is the filtered transform, then the output will be distorted. The features who have higher frequencies are located at sharp edges, and diminishing them may cause distortion.

Gaussian low-pass filters have significant roles in various applications of pattern recognition, communication, and image processing, which are categorized through bandwidths, cutoff, and overshoots, respectively. One of the important features of these filters is that the Gaussian of such filters is Gaussian as well due to which it has the same response pattern in both spatial and frequency domains, respectively, which is represented as

(10) $$\begin{array}{c} H\left(u,v\right)=e^{-D^{2}\left(u,v/2\sigma^{2}\right)}. \end{array}$$

In the frequency level at the origin, the distance is indicated by *D*(*u*, *v*); the scattering of the Gaussian curvature is calculated by *σ*. If the value of *σ* is higher, then cutoff frequency will be high. For instance, if *σ* = *r*_*0*_, then equation (10) will be re-written as

(11) $$\begin{array}{c} H\left(u,v\right)=e^{-D^{2}\left(u,v/2r_{0}^{2}\right)}. \end{array}$$

If *D*(*u*, *v*) *=* *r*_*0*_, then value of the filter is 0.671, which has the maximum value equal to 1.

A perception scheme to display an image and circular view is presented in Figure 5.

More specifically, the Gaussian low-pass filtering function for a 2D image can be written as

(12) $$\begin{array}{c} H\left(u,v\right)=e^{-u^{2}/2u_{c}^{2}}e^{-v^{2}/2u_{c}^{2}}, \end{array}$$

where *u*_*c*_ represents the cutoff frequency.

### 3.4. Signal-to-Noise Ratio (SNR)

SNR of an image is the ratio between the original intensity value and the noise. As we know that the mean of the random noise in an image is zero, thus, the SNR of the image might be measured with the help of its mean and standard deviation. Let an image be given as *C* (*x*, *y*). Therefore, the SNR of *C* (*x*, *y*) is

(13) $$\begin{array}{c} {\text{SNR}}_{C\left(x,y\right)}=\frac{\text{mean}\left(C\left(x,y\right)\right)}{\sigma_{c\left(x,y\right)}}. \end{array}$$

## 4. Performance Assessment

In order to accomplish the proposed approach, we have sequentially done the 5 × 5 averaging filter, discrete Fourier transform, and Gaussian low-pass filtering with appropriate cutoff frequency so that the SNR of the frequency domain filtered image is the same as the spatial domain image. The entire procedures are implemented in Matlab with the specification of 1.9 Hz processor and 8 GB RAM. The step-by-step procedures of the proposed approach are described as

### 4.1. Acquiring the Phantom Image

A phantom image is created with the size of 512 × 512, as shown in Figure 6.

### 4.2. Results of an Averaging Filter on the Phantom Image

As presented before, we have applied an averaging filter on the spatial domain of the image. The mask size of the filter was 5 × 5, as shown in Figure 7. Furthermore, after applying the average filter, we have obtained a smoothed image as Figure 8.

The SNR calculated for both the spatially smoothed phantom image was 37.65270.

### 4.3. Results of Discrete Fourier Transform on the Phantom Image

For such experiment, we are going to apply the frequency domain processing. In order to convert the spatial phantom image into its frequency domain, we utilized the *fft*_*2*_ function. However, after applying this function, the values of the resultant image are too high; thus, we took the log values. On the contrary, the low frequencies were at the corner that require a shifting the corner. For shifting the corner, we exploited *fft*_*2*_ function. Figures 9 and 10 demonstrate the logged image of the frequency domain representation and shifted image of the logged image. In Figure 10, the low-frequency components stay near the center, and then, it spreads out to higher frequencies.

### 4.4. Results of Gaussian Low-Pass Filter on the Phantom Image

For this experiment, we designed a rectangular low-pass Gaussian filter that takes the midposition of 512 × 512 as center. We started the cutoff frequency from 10 Hz until we get the equal and larger SNR than the spatial domain smoothed image. At last, when the cutoff frequency was 55, then we got the desired SNR and break the loop of searching the equal SNR.  Figure 11 shows the filter image with the cutoff frequency of 55.

After the first step, we multiplied the filtered image with the shifted frequency-domain transformed image. We utilized the inverse Fourier transform by *ifft*_*2*_ function against the smoothed image in order to see the filtered image in spatial domain. Hence, it gives the high-frequency removed and smoothed image, as shown in Figure 12. Moreover, Table 1 depicts the SNR for the cutoff frequency from 40 to 55.

Figure 13 shows 12 Gaussian low-pass filter images with 12 different cutoff frequencies, and Figure 14 represents the smoothing result applying the 12 different Gaussian low-pass filters shown in Figure 13.

### 4.5. Discussion

After applying the smoothing operation both in spatial and frequency domain, it is seen that the frequency domain filtering shows better smoothing than the spatial on where the SNRs are almost the same. In Figure 15, the smoothed image in frequency domain shows better edges and less noise representation than the smoothing in spatial domain. However, it may vary from time to time and depends on the types of filtering and choosing different criteria such as cutoff frequency or SNR in frequency-domain filtering. Thus, we can say that the SNR improvement of an image is very much dependent of the characteristics of the image.

Furthermore, qualitywise, the performance of the proposed approach is compared with some of the existing work [41–44] against quality measurement techniques such as SSIM, MSE, RMSE, and PSNR. The overall performance is presented in Table 2.

As can be seen from Table 1 that, after denoising, we measured the quality of the denoised images through SSIM, MSE, RMSE, and PSNR metrics. In Table 2, most of the existing methods gave consistent results against the phantom image. When the noise level increases the quality measurement matrices increase as well, the result of the proposed approach is much better than existing methods against the phantom image.

## 5. Conclusion

In medical images, noise diminishing is a challenging task for the research community in image processing. Noise produces supreme critical instabilities and degrades the quality of the medical images such as ultrasound, X-ray, and CT in healthcare. Generally, the image is considered as the collection of data and the quality of image may degrade under the presence of noises. It has to be vigorous to regenerate the noises of the original images for achieving supreme data from images. Signal-to-noise ratio (SNR) is one of the main barriers which avoids the theoretical observations to be accomplished in practice. Phantom images are generated that have well-known noises such as Gaussian noise, salt and pepper, and speckle noise. In this study, we have tried to discuss about spatial- and frequency-domain smoothing operation of a phantom image. For this purpose, several image processing methods have been utilized here such as average filtering, discrete Fourier transform, and Gaussian low-pass filtering. This work has six major parts such as applying the average filter, determining the SNR of region of interest, transforming the image in frequency domain by discrete Fourier transform, obtaining the rectangular Gaussian low-pass filter with a cutoff frequency, multiplying them, and carrying out the inverse Fourier transform. These steps are repeated accordingly until the resulting image SNR is equal to or greater than the spatial domain SNR. In order to achieve the goal of this study, we have analyzed the proposed approach against some of complex phantom images. The significances of these operators are compared against signal-to-noise ratio.

In the future research, we will deploy the proposed approach in healthcare domains such as hospitals to facilitate the physicians in various radiology domains. This approach may help the experts to accurately diagnose the corresponding disease from various radiology domains such as X-ray, CT, ultrasound, and MRI.

## Figures and Tables

**Figure 1:** The flow diagram of the proposed approach.

**Figure 2:** 3 × 3 averaging kernel commonly employed in the averaging filter.

**Figure 3:** Frequency variations of an image.

**Figure 4:** Processing of the corresponding image: (a) original image and (b) result of the FT.

**Figure 5:** Filter displayed as an image.

**Figure 6:** The overall flow of the proposed and ensembled method.

**Figure 7:** 5 × 5 averaging kernel often used in average filtering.

**Figure 8:** Smoothed image after average filtering by 5 × 5 window.

**Figure 9:** Logged frequency image of the phantom image.

**Figure 10:** Shifted image of the logged frequency image of the phantom image.

**Figure 11:** Rectangular Gaussian low-pass filter image with cutoff frequency of 55.

**Figure 12:** Smoothed image after the inverse Fourier transform of the frequency-domain filtered image.

**Figure 13:** Gaussian low-pass filter image with different cutoff frequencies.

**Figure 14:** The smoothing result using different Gaussian low-pass filters with different frequencies.

**Figure 15:** Smoothed phantom image after (a) spatial domain average and (b) frequency domain Gaussian low-pass filtering.

**Table 1:** SNR of the filtered image for the cutoff frequency from 40 to 55.

Cutoff freq.	SNR
40	35.51455
41	35.74032
42	35.95237
43	36.15139
44	36.33805
45	36.51296
46	36.67671
47	36.82986
48	36.97293
49	37.10641
50	37.23078
51	37.34648
52	37.45393
53	37.55354
54	37.64570
55	37.73075

**Table 2:** Comparison of the proposed approach with existing methods under the presence of quality measurement techniques against the phantom image (as shown in Figure 6).

Methods	Noise level	SSIM	MSE	RMSE	PSNR
[41]	0.2	0.88	19.85	13.08	22.64
	0.4	0.84	26.66	18.61	18.91

[42]	0.2	0.80	24.76	14.72	15.28
	0.4	0.90	19.01	16.99	23.05

[43]	0.2	0.85	23.89	13.91	18.89
	0.4	0.80	18.94	15.76	16.58

[44]	0.2	0.83	22.67	11.90	22.75
	0.4	0.86	18.41	14.84	18.41

Proposed approach	0.2	0.65	14.89	11.33	13.78
	0.4	0.72	15.30	12.88	16.38

## Data Availability

The data used to support the findings of the study and simulation can be obtained from the corresponding author upon request.
